# Stigmasterol alleviates cerebral ischemia/reperfusion injury by attenuating inflammation and improving antioxidant defenses in rats

**DOI:** 10.1042/BSR20192133

**Published:** 2020-04-15

**Authors:** Qilong Liang, Jun Yang, Jiaji He, Xiaoling Chen, Hong Zhang, Maolin Jia, Kai Liu, Chuangchuang Jia, Yanhong Pan, Jinwang Wei

**Affiliations:** Department of Neurosurgery, Second Hospital of Lanzhou, Lanzhou City 730046, Gansu Province, P.R. China

**Keywords:** cerebral ischemia/reperfusion (I/R) injury, inflammation, oxidative stress, stigmasterol

## Abstract

***Background/aims:*** The paper aimed to investigate the effects of Stigmasterol on inflammatory factors, antioxidant capacity, and apoptotic signaling pathways in brain tissue of rats with cerebral ischemia/reperfusion (I/R) injury. ***Methods:*** The neurological deficits of the rats were analyzed and HE staining was performed. The cerebral infarct volume was calculated by means of TTC staining, and neuronal apoptosis was detected by TUNEL staining. At the same time, the contents of glutathione peroxidase, glutathione, superoxide dismutase (SOD), nitric oxide, and malondialdehyde in brain tissue were measured. The expression of the relevant protein was detected by means of Western blotting. ***Results:*** The results showed that the neurological deficit score and infarct area of the I/R rats in the soy sterol treatment group were significantly lower than those in the I/R group. Moreover, the levels of carbon monoxide and malondialdehyde in the soysterol group were significantly lower than those in the I/R group, and the expressions of cyclooxygenase-2 (Cox-2) and NF-κB (p65) in the soysterol group were also significantly lower than those in the I/R group. The expression of Nrf2 (nucleus) and heme oxygenase-1 (HO-1) increased significantly, and the activities of antioxidant enzymes and SOD were increased. In addition, the stigmasterol treatment can inhibit apoptosis, down-regulate Bax and cleaved caspase-3 expression, and up-regulate Bcl-Xl expression. ***Conclusion:*** Stigmasterol protects the brain from brain I/R damage by reducing oxidative stress and inflammation.

## Introduction

Cerebrovascular disease has become an important disease causing death, with high morbidity, mortality, and disability [1,2]. Cerebral infarction refers to the supply of blood flow to the brain caused by various causes, causing irreversible damage to the brain tissue. It leads to ischemia and hypoxic necrosis of the brain tissue, which is a common hazard to human health. The reduction in cerebral blood flow is the most common cause of irreversible brain damage [3]. Early recovery of cerebral blood perfusion, oxygen supply to ischemic brain tissue, nutrients necessary for metabolism, and removal of metabolic waste are helpful to alleviate cerebral ischemic injury and functional recovery of some reversible injuries. It is the fundamental measure to alleviate ischemic brain injury [4]. However, studies have found that recovery of blood flow after ischemia can lead to further tissue damage and dysfunction in some cases. This regenerative condition after restoring blood perfusion is called ischemia/reperfusion (I/R) injury. Ischemic brain injury includes primary injury during ischemia and secondary injury during reperfusion, and re-injury to restore blood perfusion of brain tissue is inevitable [5,6]. Exploring the mechanism of brain injury and finding drugs to alleviate cerebral ischemia and reperfusion injury has become the focus of cerebral ischemia treatment.

Traditional Chinese medicine plays a unique role in this respect, mainly in antioxidant and pathological damage, reducing neurotoxins of excitatory amino acids, scavenging free radicals, reducing calcium overload, affecting platelets and thrombosis, gene expression, and apoptotic regulation. Stigmasterol is the main plant sterol in various herbs and has strong pharmacological activity [7,8]. A schematic diagram of the structure of stigmasterol was shown in Figure 1A. Studies have shown that stigmasterol can significantly improve heart and cerebral I/R injury. Its role includes reducing infarct size, increasing the activity of superoxide dismutase (SOD) in myocardium and plasma, scavenging oxygen free radicals, calcium antagonism, improving microcirculation, reducing brain water content, calcium ions, glutamic acid, aspartic acid, glycine, and lipid peroxidation product malondialdehyde in rats with I/R. However, the mechanism of action of stigmasterol is not fully disclosed.

**Figure 1:** The investigation of Stigmasterol in cerebral ischemia/reperfusion injury (**A**) Stigmasterol (chemical formula of C_29_H_48_O with a molecular weight of 412.69). (**B**) Schematic diagram of the experimental protocol.

In the present study, the rat middle cerebral artery occlusion reperfusion model was used to observe the expression of stigmasterol after I/R and its effect on inflammatory and antioxidant factors in brain tissue. It will provide some valuable information for further exploring the mechanism of cerebral I/R injury and brain protection mechanism.

## Materials and methods

### Experimental animal

Wistar rats supplied by the Laboratory Animal Center of Second Hospital of Lanzhou are magnetic. Their weight ranges from 185 to 225 g. All experiments were performed in the Laboratory Animal Research Center of Second Hospital of Lanzhou and they were approved by Second Hospital of Lanzhou Ethical Committee before the experiment.

### Focal cerebral I/R model

Wistar rats were randomly divided into four groups: sham operation group, I/R model group, I/R model + stigmasterol 20 mg.kg^−1^ group, blood reperfusion model + stigmasterol 40 mg.kg^−1^ group, and blood reperfusion model + stigmasterol 80 mg.kg^−1^ group. According to the test results, the doses of stigmasterol used in the study were 20, 40, and 80 mg/kg, respectively. After 1 week of administration, the model group and the sham group were equal to the same amount of normal saline. After the last administration of anesthesia, the MCAO model was prepared according to the reference [9]. Through the main incision of external carotid artery, nylon thread was slowly pushed to the direction of internal carotid artery entering the skull to reach a smaller anterior cerebral artery and block all blood supply of middle cerebral artery (MCA). Focal cerebral I/R model was according to literature [9]. The specific experimental design of the study was shown in Figure 1B.

### Neurological assessment

After 300 min of MCAO, Longa method was used to evaluate the neurobehavioral status of animals.

### Determination of infarct volume

Five hours after MCAO, the rats were killed by decapitation. The whole brain was taken out, the left and right brains were separated. The right brain was taken out, and the cerebellum, lower brainstem, and olfactory bulb were removed. Then the wet weight was weighed immediately. The right forebrain was then cut along the coronal plane and brain sections were placed in 1.5 ml of 2% TTC solution and kept in the dark for 30 min. Brain sections were then fixed with 10% formaldehyde. The pallorous area (infarct area) and the non-pallord area (normal area) were separated by ophthalmology, and the percentage of infarction was calculated by literature. Percentage of infarction (%) = weight of pale area/(weight of pale area + weight of non-pallord area) × 100%.

### HE dyeing

After deep anesthesia, the rats were perfused with normal saline and 40 g/l paraformaldehyde fixative, and stored in 200 g/l sucrose overnight. Coronal sections of 30 micron brain tissue were made by frozen section machine at 2 mm after optic chiasm, and 10–15 micron sections of adjacent tissues were made for HE staining.

### Determination of antioxidant index

Five hours after MCAO, the rats were killed by decapitation. The blood was treated by centrifugation, the supernatant in the blood was aspirated into a centrifuge tube, and it was chilled at a temperature of 4°C. The right hemisphere was cut from frontal pole to occipital lobe, and the occipital lobe was homogenized in frozen saline. The contents of NO (Griess method), SOD (enzyme labeling method), MDA (thiobarbituric acid method), GSH (colorimetric method), and GSH-Px (colorimetric method) in brain tissue and serum were determined.

### TUNEL staining

The TUNEL staining was used to detect cell apoptosis on the basis of DNA fragmentation that results from the apoptosis-signaling cascades. The brain (*n*=6) was examined after 24-h reperfusion with sodium chloride and 4% formaldehyde, regularly embedded in paraffin and was then sectioned at a thickness of 4 μm. TUNEL staining was performed according to the manufacturer’s instructions (Roche Diagnostics Corp., Indianapolis, U.S.A.) for the TUNEL assay kit. The total number of cells and the number of TUNEL-positive cells was observed under a light microscope (Olympus BX51; Olympus Co., Tokyo, Japan). Five high-power fields of the ischemic cerebral penumbra areas were randomly selected, and the number of apoptotic cells for each field was counted. The apoptosis index (AI) = the number of positive cells/the number of total cells.

#### Western blot

After the 24-h reperfusion, the rat brains were removed and stored at −80°C until use. The brains (*n*=6) were gently homogenized in lysis buffer (1.5 mmol/l MgCl_2_, 10 mmol/l KCl, 20 mmol/l HEPES, 1 mmol/l EDTA, 1 mmol/l EGTA, 250 mmol/l sucrose, 0.1 mmol/l phenylmethylsulfonyl fluoride (PMSF), 1 mmol/l dithiothreitol (DTT), and proteinase inhibitor cocktail; pH 7.9). The tissues were centrifuged at 14000 rpm at 4°C for 15 min. The supernatant was collected and assayed for the determination of the total protein concentrations using the Bradford assay with bovine serum albumin (BSA) as the standard. The nuclear extraction was performed according to the method described previously. Briefly, the brain tissue was homogenized in an ice-cold hypotonic lysis buffer containing 10 mM HEPES (pH 7.9), 1.5 mM magnesium chloride (MgCl_2_), 10 mM potassium chloride (KCl), 0.5 mM PMSF, 0.5 mM DTT, a protease inhibitor, and 1% NP-40. Then, the homogenate was centrifuged at 13000 rpm for 30 s at 4°C. The nuclear pellet was resuspended in an ice-cold hypertonic extraction buffer containing 10 mM HEPES (pH 7.9), 0.42 M NaCl, 1.5 mM MgCl_2_, 10 mM KCl, 0.5 mM PMSF, 1 mM DTT, and protease inhibitors at 4°C for 30 min. After centrifugation at 14000 g for 5 min, the nuclear extract was collected, and the protein concentrations were determined by using the Bradford protein assay. Equal amounts of protein were separated on a 10 ± 15% SDS/polyacrylamide gel and were then transferred to a PVDF membrane (Immobilon-P, Millipore, Bedford, MA, U.S.A.) at 400 mA for 35 min. After blocking with 5% skim milk in TBS containing 0.1% Tween-20 (TBST) at 4°C for 3 h, the membrane was incubated with primary antibodies anti-Bax (1:1000; ab32503, Abcam, Cambridge, MA); anti-Bcl-XL (ab32370; Abcam, Cambridge, MA); anti-caspase-3 (ab13847; Abcam, Cambridge, MA); anti-Nrf2 (ab31163; Abcam, Cambridge, MA); anti-HO-1 (ab137749; Abcam, Cambridge, MA); anti-p65 (ab16502; Abcam, Cambridge, MA); anti-Cox2 (ab52237; Abcam, Cambridge, MA); anti-GAPDH (ab128915; Abcam, Cambridge, MA); HRP-conjugated goat anti-rabbit IgG, ab205718; Abcam, Cambridge, MA, U.S.A.) were added. After incubation overnight, 1:5000 labeled anti-rabbit secondary antibody was added. Then the Western blot analysis was carried out according to Literature [10].

### Statistical method

With the help of SPSS software, statistical analysis of the data obtained is carried out, and the results of data analysis are expressed by the mean (+standard deviation). Multigroup data analysis is based on one-way ANOVA. LSD testing is used for subsequent analysis. *P*<0.05, the results have significant difference.

## Results

### Stigmasterol can alleviate the neurological deficit and infarct volume of stroke rats to a certain extent

Neurological deficits 24 h after reperfusion were scored, and the results were shown in Figure 2A. From the experimental results, we can know that the neurological deficit score in the I/R group was significantly higher than that in the sham operation group (*P*<0.01). The scores of neurological deficits in the different doses of stigmasterol group were significantly lower than those in the I/R group (*P*<0.05, *P*<0.01).

**Figure 2:** Effect of stigmasterol on neurological behavioral scores and cerebral infarction volume after I/R in rats (**A**) Neurological deficit score after brain I/R. (**B,C**) TTC staining of coronal brain sections 24 h after reperfusion. (**D,E**) TTC staining of coronal brain sections at 2, 12 and 48 h after reperfusion. *P<0.05, **P<0.01 vs the sham operation group. ^##^*P* <0.01 vs I/R group.

Stroke-size TTC staining showed that the percentage of infarct volume in the I/R group was significantly higher than that in the sham-operated group (*P*<0.01). The percentage of infarct size in the different stigmasterol dose groups was significantly lower than that in the I/R group (*P*<0.05, *P*<0.01) (Figure 2B,C). In addition, to study the infarct volume of MCAO+80 mg/kg stigmasterol group and MCAO+carrier group at different time after reperfusion (Figure 2D,E), there was no difference between MCAO+80 mg/kg stigmasterol group and carrier group. Compared with the vehicle-treated group, the percentage of 80 mg/kg stigmasterol infarct volume was significantly decreased at 12 and 48 h after reperfusion (*P*<0.05, *P*<0.01).

### Stigmasterol reduced the neuronal loss in hippocampus following I/R

Here, the effects of stigmasterol on neuronal morphologic damage in stroke rats were evaluated by H&E staining (Figure 3A). The number of intact neurons were counted, and the results showed that the brain of the stigmasterol treatment groups decreased the number of degenerated neurons, and the number of normal neurons increased in the ischemic penumbra cortex. For the morphologic change, the brain sections of the normal (sham) group remained intact and with normal cell organelles, the neurons were still arranged well, and the nuclei were centered with clear staining, whereas the vehicle (I/R) group showed many vacuolated spaces and neuronal loss. From Figure 3B, we can see that the number of hippocampal neurons in the stigmasterol group was significantly higher than that in the I/R group (*P*<0.05, *P*<0.01).

**Figure 3:** Protective effects of stigmasterol on hippocampal neurons (**A**) Cerebral ischemia-hippocampal staining after reperfusion arrows (thin arrow, intact cells; thick arrow, damaged cells). (**B**) Statistical results of surviving neurons in each group. *P<0.05, **P<0.01 vs the sham operation group; ^##^*P*<0.01 vs the I/R group.

### Stigmasterol reduced lipid peroxidation in stroke rats

From the results of Figure 4, compared with sham-operated group, the level of MDA in the brain of group R was significantly higher (*P*<0.01). The MDA level of rats in different stigmasterol groups was significantly lower than that in I/R group (*P*<0.05, *P*<0.01).

**Figure 4:** Stigmasterol reduced markers of lipid peroxidation in the ischemic tissue *P<0.05, **P<0.01 vs the sham operation group; ^##^*P*<0.01 vs the I/R group.

### Stigmasterol can relieve inflammation to a certain extent and promote the improvement of antioxidant capacity in tissues

As shown in Figure 5A–C, compared with the sham operation group, the expression levels of COX-2 and NF-κB (p65) in the I/R group were significantly higher (*P*<0.01), while stigmasterol (40 and 80 mg/kg) significantly inhibited the expression of NF-κB (p65) and cyclooxygenase-2 (Cox-2) (*P*<0.01). In addition, from the results of NO content analysis in the brain, we can know that compared with the sham operation group, the NO content in the I/R group was significantly higher (*P*<0.01). Different doses of stigmasterol significantly reduced NO levels in a dose-dependent manner (*P*<0.05, *P*<0.01) (Figure 5D).

**Figure 5:** Inflammation of brain I/R rats is affected by myristyl alcohol (**A**) Cox-2 and NF-κB (p65) protein expression levels. (**B**) Quantitative results of NF-κB (p65) protein expression. (**C**) Quantitative results of COX-2 protein expression. (**D**) No grade. *P<0.05, **P<0.01 vs the sham operation group; ^##^*P*<0.01 vs the I/R group.

We can see from Figure 6A-C that the expression levels of nrf2 protein and heme oxygenase-1 (HO-1) protein in the nucleus of the I/R group were significantly lower than those in the sham operation group (*P*<0.01), while the expression of Nrf2 protein and HO-1 protein in the nucleus of different stigmasterol doses groups was significantly increased (*P*<0.05, *P*<0.01). From the results, we can know that stigmasterol can promote the antioxidant capacity of the tissue to a certain extent. From Figure 6D–F, we can see that the levels of SOD, GSH, and GSH-Px in the I/R group were significantly lower than those in the sham-operated group (*P*<0.01), while the different doses of the stigmasterol group. The levels of GSH-Px, GSH, and SOD were significantly higher (*P*<0.05, *P*<0.01). These results indicated that stigmasterol enhanced the tissue’s antioxidant defense ability by activating the Nrf2 signaling pathway.

**Figure 6:** Effect of stigmasterol on Nrf2 signaling pathway in rat brain with I/R injury (**A**) Nrf2 (nucleus) and HO-1 protein expression levels. (**B**) Quantitative results of Nrf2 protein expression in each group. (**C**) Quantitative results of HO-1 protein expression. (**D**) SOD activity. (**E**) Content of GSH. (**F**) Content of GSH-Px. *P<0.01, **P<0.01 vs the sham operation group, ^##^*P*<0.01 vs the I/R group.

### Stigmasterol treatment reduced apoptotic markers in the ischemic tissue

The experimental results are shown in Figure 7. From the figure, we can see that the expression levels of cleaved caspase-3 and bax in the I/R group were significantly higher than those in the sham operation group, while the expression level of bcl-Xl was significantly lower than that in the sham operation. In the group (*P*<0.01), the expression level of bcl-Xl in the I/R group was much lower than that in the sham operation group (*P*<0.01).

**Figure 7:** Effect of stigmasterol on I/R-induced apoptosis in rat cells (**A**) Expression of Bax, Bcl-Xl, and cleaved caspase-3 protein in rat brain tissue. (**B**) Quantitative results of Bcl-Xl protein expression in each group. (**C**) Quantitative results of Bax protein expression in each group. (**D**) Quantitative results of expression of cleaved caspase-3 protein in each group. *P<0.05, **P<0.01 vs the sham operation group; ^##^*P*<0.01 vs the I/R group.

From Figure 7A–D, we can see that the expression levels of cleaved caspase-3 and Bax after treatment with stigmasterol are much lower than those in I/R group, while bcl-Xl protein level is very large. The degree was higher than the I/R group (*P*<0.05, *P*<0.01). By means of TUNEL staining, we can see that there are only a few TUNEL-positive cells in the sham operation group, and the number of TUNEL-positive cells in the I/R group is significantly higher than that in the sham-operated group (*P*<0.01). The number of TUNEL-positive cells in the different doses of stigmasterol treatment group was significantly reduced compared with that in I/R group (*P*<0.05, *P*<0.01) (Figure 8). These results indicated that stigmasterol had an anti-apoptotic effect on I/R injury.

**Figure 8:** Effect of stigmasterol on I/R-induced apoptosis in rat cells Arrows were used to indicate cells that presented characteristic morphological changes of apoptosis. *P<0.05, **P<0.01 vs the sham operation group; ^##^*P*<0.01 vs the I/R group.

## Discussion

Stroke is a group of acute cerebrovascular diseases with symptoms of cerebral ischemia and hemorrhagic injury as the main clinical manifestations [11,12]. The brain has complex functions but almost no energy reserves, and is poorly tolerant to ischemia and hypoxia, requiring blood circulation to continuously supply oxygen and glucose. Cerebral blood vessels have a strong autoregulatory function, but ischemic brain damage occurs when cerebral blood flow is reduced until the transport of metabolites is insufficient to meet metabolic needs. The central problem of cerebral ischemia is the depletion of oxygen and energy. Therefore, increasing the supply of oxygen and blood in ischemic brain tissue early in the time window is the key to the prevention and treatment of ischemic brain injury [13,14]. Previous studies have found that stigmasterol effectively depressed the expression level of beclin1, and the conversion of LC3 I into LC3 II, while promoted the phosphorylation of mTOR, and remarkably inhibited the phosphorylation of AMPK and JNK, as well as the expression of JNK [15]. In our study, stigmasterol alleviates cerebral I/R injury by attenuating inflammation and improving antioxidant defenses in rats by NF-κB p65 pathway. The experimental results showed that after reperfusion, stigmasterol can reduce the infarct size and the neurological deficit, alleviate the pathological changes caused by ischemia, and these results are basically the same with the literatures.

Oxidative stress is one of the most important pathological mechanisms of ischemic stroke [16]. Nrf2 belongs to the leucine zipper family. It is an important transcription factor regulating the oxidative stress [17,18]. In the case of oxidative stress, Keap1 dissociates from Nrf2, and Nrf2 undergoes nuclear translocation into the nucleus and binds to the antioxidant response element (ARE) [19,20]. ARE-regulated antioxidant proteins includes HO-1, GST, GSH etc., which can protect the body from reactive oxygen species [21]. In animal experiments, cell *in vitro* experiments and Nrf2 gene knockout experiments, it has been confirmed that Nrf2 knockout in mice increases cerebral ischemic injury, activates Keap1/Nrf2/ARE pathway, promotes the expression of HO-1 and other proteins, and alleviates cerebral ischemic injury [22]. This study found that the expression of Nrf2 and HO-1 protein in the nucleus of the stigmasterol-treated rats was significantly increased. Stigmasterol further activated Nrf2/ARE signaling pathway, promoted the synthesis and nuclear translocation of Nrf2 protein. The chain reaction induced by reactive oxygen species is the core pathological part of brain tissue I/R injury. Excessive oxygen free radicals cause neuronal necrosis or apoptosis in brain tissue through many links [23]. MDA can reflect the degree of vascular damage and the level of oxygen free radicals present [24]. As a free radical scavenger, SOD, CAT, GSH, and GSH-Px have significant antioxidative effects in cerebral ischemia and hypoxia, and have received increasing attention [25,26]. The results showed that the activities of GSH-Px, GSH, CAT, and SOD in brain tissue of rats with cerebral I/R injury decreased to a large extent, while the content of malondialdehyde increased to some extent. Stigmasterol can significantly inhibit the decrease of SOD, CAT, and GSH-Px and the increase in MDA in serum and brain tissue of model rats. It indicated that after cerebral ischemia and reperfusion, the free radical production in brain tissue increased, and a significant lipid peroxidation reaction occurred. Stigmasterol can reduce the production of free radicals and lipid peroxidation, which showed good antioxidative damage.

The expression of NF-κB p65 mRNA and protein was significantly increased in ischemic brain tissue. Inhibition of NF-κB expression reduced cerebral infarction area and neuronal death in MCAO rats [27]. Among these neuroinflammatory events, those elicited through NF-κB p65 play an important role in the induction of excessive production of inflammatory factors and ischemic brain damage, as evidenced by previous studies showing that downstream NF-κB p65 protects the brain from ischemic damage and neurodegeneration in MCAO rats [28]. This study found that the expression of NF-κB p65 in the model group was significantly increased, indicating that NF-κp p65 was activated and translocated into the nucleus. Stigmasterol significantly reduced the expression of NF-κB p65, indicating that it blocked activation of NF-κB. As a downstream target gene of NF-κB, iNOS, and Cox-2 are rapidly induced to express under cerebral ischemia, and they coordinate with each other to directly damage the DNA and protein of the cells [29]. Cox-2 is an inducible cyclooxygenase, a marker of inflammatory response and a key enzyme in neuronal death caused by cerebral ischemia [30]. iNOS is induced by macrophages, neuroglia, neurons etc., after stimulation of cerebral ischemic injury. Once formed, a large amount of NO is slowly and permanently produced, resulting in apoptosis of nerve cells [31]. Studies showed that the expression of iNOS, Cox-2, and NF-κB in brain tissue of MCAO model mice was up-regulated after 2 h of ischemia. At the same time, a large number of free radicals were released, which destroyed the blood-brain barrier, enlarged the area of cerebral infarction and severely damaged neurons [32]. The results showed that the levels of NO and COX-2 of the model group were significantly increased, suggesting that COX-2 and NO were involved in cerebral I/R injury. Stigmasterol can significantly reduce NO levels and COX-2 expression and reduce the nerve damage it mediated.

The relationship between pro-apoptotic genes (such as Bax) and anti-apoptotic genes (such as Bcl-XL) is an important factor in determining whether cells undergo apoptosis and the severity of apoptosis [33]. Recent studies have shown that the caspase family plays a key role in ischemic injury. Caspase-3 is the only way to cascade activation, and is at the core. It is also known as death protease, which plays a final pivotal role in the apoptotic program initiated by various factors [34]. In the nervous system, caspase-3 can not only promote the apoptosis of neurons during brain development, but also promote the apoptosis of cultured neurons induced by various factors [35]. This study found that after stigmasterol treatment, the expression of Bax and caspase-3 were significantly decreased, Bcl-Xl protein levels were increased significantly, and apoptosis rates were increased significantly. Stigmasterol had protective effects on cerebral I/R injury, which may be achieved mainly by reducing proapoptotic genes (Bax), caspase-3 and increasing anti-apoptotic genes (Bcl-XL).

## Conclusion

Stigmasterol can relieve oxidative stress, inflammation, and apoptotic responses to a certain extent to protect the brain from brain I/R damage.

## Abbreviations

ARE: antioxidant response element
Cox-2: cyclooxygenase-2
DTT: dithiothreitol
HO-1: heme oxygenase-1
I/R: ischemia/reperfusion
Keap1: kelch like ECH associated protein 1
MCAO: middle cerebral artery occlusion
nrf2: nuclear factor E2-related factor 2
PMSF: phenylmethylsulfonyl fluoride
SOD: superoxide dismutase
